# Study on the Mechanism of Shenjing Guben Prescription Regulating PI3K and NRF2 Signaling Pathway in the Treatment of Immune Infertility

**DOI:** 10.1155/2022/8754188

**Published:** 2022-05-13

**Authors:** Handu Liu, Jianguo Xue, Hui Mo

**Affiliations:** ^1^Faculty of Chinese Medicine, Macau University of Science and Technology, Wai Long Avenue, S.A.R. 999078, Taipa, Macau; ^2^Andrology, Affiliated Hospital of Nanjing University of Chinese Medicine, Nanjing, China

## Abstract

**Objective:**

To explore the mechanism of Shenjing Guben prescription (SP) in the treatment of immune infertility by regulating PI3K-NRF2/p38 signal pathway.

**Methods:**

60 adult male SD rats were randomly divided into control group (NC group), ACN group, low concentration AP intervention group (low group), middle concentration SP intervention group (middle group), and high concentration SP intervention group (high group). 12 rats in each group were administered by gavage once a day, 6 days/w, and the rats were killed after 28 days. Bilateral testis and epididymis were removed and weighed and organ coefficients were calculated, and testicular histopathological sections were prepared to evaluate the changes of testicular tissue structure. The relative expression levels of PI3K, MKK7, JNK, p38 mRNA, and protein in testis were measured by QRT-PCR and western blot.

**Results:**

(1) Compared with the control group, the proportion of grade A and B sperms in ACN group increased significantly, and the proportion of grade D sperm decreased significantly (*P* < 0.05). After SP intervention, compared with ACN group, there was no significant difference in the proportion of sperm at all levels in low, medium, and high SP intervention groups (*P* > 0.05). (2) Compared with the control group, the sperm VCL, VSL, VAP, and mad in ACN group increased significantly, and the BCF decreased significantly (*P* < 0.05). After SP intervention, compared with ACN group, there was no significant difference in sperm motility parameters among low, medium, and high SP intervention groups (*P* > 0.05). (3) Compared with the control group, the activities of AKP and SDH in testicular tissue of rats in ACN group decreased significantly (*P* < 0.05). After SP intervention, compared with ACN group, AKP activity increased significantly and LDH activity decreased significantly in low, medium, and high SP intervention groups (*P* < 0.05). (4) Compared with the control group, the expression levels of PI3K, p-PI3K, MKK7, p-MKK7, JNK, p-JNK, p38, and p-p38 proteins and the ratios of p-JNK/JNK and p-p38/p38 increased in the testis of ACN group (*P* < 0.05). After SP intervention, compared with ACN group, the protein expression levels of PI3K, p-PI3K, MKK7, p-MKK7, JNK, p-JNK, p38, and p-p38 in testicular tissue of SP intervention group decreased, and the ratio of p-JNK/JNK and p-p38/p38 decreased (*P* < 0.05).

**Conclusion:**

SP can reduce the oxidative stress of testis induced by ACN and inhibit the activation of PI3K-NRF2/p38 signal pathway.

## 1. Introduction

Acrylonitrile (ACN), also known as ethylene cyanogen, is a colorless, flammable, volatile liquid with bitter almond flavor. ACN is an important organic chemical synthetic monomer. It is an important raw material for manufacturing synthetic resin, synthetic rubber, synthetic plastics, synthetic fiber, and acrylamide [1]. ACN can also be detected in cigarette smoke and automobile exhaust. Therefore, low-dose environmental exposure cannot be ignored. ACN and CEO can also combine with biological macromolecules such as protein or DNA to consume GSH in tissues. The depletion of GSH will reduce the antioxidant capacity of the body, and cytochrome P450 metabolizing ACN can produce more free radicals in the metabolic process, further increasing the load of oxidative stress. ACN is a highly toxic compound. It is a mutagen and suspected carcinogen in humans. Its exposure will increase the risk of lung cancer and astrocytoma [2].

Traditional Chinese medicine recognizes that kidney deficiency and blood stasis are the fundamental pathogenesis throughout the whole process. The basic guiding principle of clinical treatment is the method of kidney activating blood circulation. Based on many years of clinical practice experience and the principle of kidney tonifying method, traditional Chinese medicine is committed to the clinical and basic research of kidney tonifying and blood activating traditional Chinese medicine in the treatment of sperm deficiency infertility. Shenjing Guben prescription consists of pilose antler, cinnamon, red ginseng, *Astragalus membranaceus*, *Rehmannia glutinosa*, polygonatum, *Polygonum multiflorum*, *Cornus officinalis*, raspberry, etc. SP can upregulate the expression of Caspase-7 in spermatozoa and inhibit the function of spermatozoa. Ginseng pill can protect spermatozoa by upregulating the expression of Caspase-7 in spermatozoa. However, the overactivation of primitive spermatheca is an important pathological mechanism leading to dor. PI3K-jnk/p38 signal pathway is to maintain the primitive spermatozoa in the static state of bubbles, and the initiation of supplementary growth is an important regulatory factor. In the dormant state of primitive spermatozoa, the activity is inhibited. Once the signal is activated, the primitive spermatozoa will be activated, growth into the vesicle pool of sperm. Granulosa cell apoptosis is the central link in the induction of sperm atresia. PI3K-jnk/p38 signaling pathway plays a key regulatory role in the apoptotic pathway. Oxidative stress is an important factor to start the apoptotic process. The essence of apoptosis is the result of the destruction of the dynamic balance between intracellular oxidation system and antioxidant system. PI3K-jnk/p38 signal pathway is the most important endogenous antioxidant stress signal pathway found so far, which is of great significance to maintain the normal growth and development of sperm [3]. Gutierrez et al. found that SP can protect mouse cardiomyocytes from injury induced by lipoteichoic acid by inhibiting the activation of JNK and p38 [4]. Zhang et al. found that SP can improve the decrease of SOD and GSH PX activity and the increase of MDA content, downregulate the expression of Caspase-3 and Bax, upregulate the expression of Bcl-2, show antioxidant and antiapoptotic characteristics, and promote the recovery of neural function in rats after spinal cord injury [5]. Dang et al. found that SP can downregulate the expression of Caspase-3, suggesting that SP can inhibit germ cell apoptosis and reduce the inflammatory response caused by ACN by downregulating NF signal [6]. Li et al. [7]. found that SP can reduce inflammatory factors in mouse lung tissue, prevent the phosphorylation of p38 and JNK, upregulate the expression of Bcl-2, and downregulate the expression of Bax and Caspase-3, suggesting that SP can play a protective role in LPS induced acute lung injury by reducing inflammatory response, inhibiting p38 MAPK and JNK signaling pathway and apoptosis [8]. Lin et al. found that SP inhibited dopamine-induced melanocyte apoptosis by reducing the production of ROS and inhibiting the activation of JNK and p38 MAPK signaling pathways [9].

## 2. Method

### 2.1. Experimental Animals

There were 60 adult male SD rats, weighing 180∼220 g. The experiment was approved by the ethics committee of our hospital. Sixty male SD rats were randomly divided into five groups with 12 rats in each group according to their body weight: control group (NC group), ACN group, low concentration SP intervention group (low group), medium concentration SP intervention group (middle group), and high concentration AP intervention group (high group). ACN and AP were prepared into the required dose with corn oil and were administered by gavage according to the gavage amount of 5 ml/kg. The gavage amount was adjusted by weighing every two days. Low, medium, and high SP intervention groups were given ACN 30 minutes after SP gavage. Once a day for 28 consecutive days, the dose selection of ACN was determined according to the previous study. SP showed antioxidant effect in rat testicular tissue in the range of 234∼468 mg/kg. Therefore, this study established the model of reproductive injury induced by ACN by 46 mg/kg ACN for 28 days and intervened with 117, 234, and 351 mg/kg SP at the same time. The feeding temperature is 21∼24°C, and the relative humidity is 40%∼60%. The laboratory is illuminated day and night for 12 hours. It is fed with ordinary feed and can eat and drink freely.

### 2.2. Sperm Density

Select the left epididymis of 6 rats in each group, cut 3 openings laterally in the epididymis, put it into an ampoule containing 0.9% normal saline, bathe in water at 37°C for 50 minutes, and suck sperm suspension for 10 minutes. It was added to the sperm counting plate and determined by computer-aided sperm analysis (CASA). The following parameters were measured: (1) sperm density: the number of sperm per ml of semen (×10^6^/ml). (2) Sperm motility and mobility: sperm can be divided into four grades according to different movement modes: grade A sperm is fast linear forward moving sperm, and straight fine velocity (VSL) ≥25 *μ*m/s; grade B spermatozoa are slow or nonlinear forward motile spermatozoa with VSL ranging from 5 to 25 *μ*M S; grade C sperms are nonforward motile sperm with VSL <5 *μ*m/s; grade D sperms are immobile sperm. (3) Sperm viability refers to the percentage of “a + B + C” sperm in semen. (4) Sperm motility refers to the percentage of “a + B” sperm in semen.

### 2.3. Determination of Testicular Tissue Marker Enzymes

Take the right testis of 8 rats in each group, cut 100∼200 mg and put it into the glass homogenizer. Add precooled 0.9% normal saline according to the ratio of tissue (g): homogenization medium (ML) = 1 : 9, grind it fully in ice water bath, centrifuge at 2500 rpm for 10 min, absorb the supernatant, and prepare 10% testicular tissue homogenate. Detect the activities of alkaline phosphatase (AKP), acid phosphatase (ACP), succinate dehydrogenase (SDH), and lactate dehydrogenase (LDH) according to the steps on the instructions of the kit.

### 2.4. Determination of Oxidative Stress-Related Indexes

Take 10% testicular tissue homogenate and determine the contents of GSH and MDA and the activities of SOD, GSH PX, and catalase (CAT) according to the operation steps on the manual. Take the right testicular tissue of rats with the same number, add precooled 0.9% normal saline according to the ratio of testicular tissue (g): homogenate medium (ML) = 1 : 4, grind in ice water bath to obtain 20% testicular tissue homogenate, centrifuge at 12000 rpm for 5 min, and absorb the supernatant to detect the total antioxidant capacity (T-AOC).

### 2.5. RT-PCR

RT-PCR was used to detect the mRNA expression of PI3K, MKK7, p38, JNK, Bax, and Bcl-2 in testicular tissue. Total testicular RNA was extracted with Trizol reagent. According to the supplier's instructions, use the primescript first strand cDNA synthesis kit from 2 *μ*l total RNA synthesis cDNA. Use SYBR premix ex Taq *μ* II kit and 10 *μ*l SYBR premix ex Taq for ™ II kit for real-time quantification ™ The expression level of the gene was normalized to *β*- The expression level of actin mRNA. Real-time polymerase chain reaction was performed using an applied biological system type 7500. The reaction conditions are 95°C 5 min, 95°C 30 s, 63°C 50 s, 72°C 60 s, 30 cycles, and 72°C 5 min. The relative expression of the target gene is calculated by 2^−∆∆CT^.

### 2.6. Protein Expression Was Detected by Western Blot

Total tissue protein was extracted and quantified by BCA protein analysis kit. Total protein was isolated by 10% SDS-PAGE (20 *μ*g) and it was transferred to polyvinylidene fluoride (PVDF) membrane. 5% skimmed milk powder was dissolved in Tris buffer solution containing 0.1% Tween 20 for blocking and then incubated with MKK7, p-MKK7, p38, p-p38, JNK, p-JNK, and Caspase-9 antibodies at 4°C overnight. On the 2nd day, the membrane was washed with PBS for 3 times, and the Goat antirabbit IgG antibody coupled with horseradish peroxidase (HRP) was incubated at room temperature for 1 h. Add an appropriate amount of ECL light solution in the darkroom for development and fixation. After scanning the strip, analyze the gray value with ImageJ software to calculate the relative expression of protein.

### 2.7. Apoptosis of Rat Testicular Cells Was Detected by TUNEL Method

Take rat testicular tissue sections for dewaxing and hydration; hydrogen peroxide is treated at room temperature for 10 min and washed with water; after incubation with protease K diluted with 0.01 mol/L TBS 1 : 200 at 37°C for 10 min, rinse with 0.01 mol/L TBS for 3 times for 5 min each time; take 1 TDT and 1 dig-d-utp respectively *μ* 50. Add 18 *μ*l labeling buffer, mix well, add it to the slices, incubate at 37°C for 2 hours, and rinse with 0.01 mol/L TBS for 3 times for 5 minutes each time; plus 50 *μ* L blocking solution, incubate at 37°C for 30 min and throw off the blocking solution; add biotinylated antidigoxin antibody diluted 100 times with antibody diluent and react at 37°C for 30 min. Rinse 3 times with 0.01 mol/L TBS for 5 min each time; SABC diluted 100 times with antibody diluent was added. After reacting at 37°C for 30 min, 0.01 mol/L TBS was rinsed for 4 times for 5 min each time; take one drop of A, B, and C in DAB kit, add 1 ml deionized water, mix well, add it to the slice for color development, and wash with water; hematoxylin is lightly counterstained, washed, dried, and sealed.

### 2.8. Statistical Analysis

SPSS 20.0 and GraphPad Prism 5.0 software were used for data processing. The measurement data were expressed by mean ± standard deviation, one-way ANOVA was compared among multiple groups, and LSD test was used for pairwise comparison. *P* < 0.05, the difference was considered to be statistically significant.

## 3. Results

### 3.1. General Conditions and Organ Coefficient Changes of Rats

During the experiment, the rats in ACN group showed salivation, and irritability in the second week, and no abnormal behavior was observed in other groups. There was no significant difference in body weight between groups before the experiment (*P* > 0.05). After the experiment, there was no significant difference in testicular wet weight and testicular organ coefficient between groups (*P* > 0.05). Compared with the control group, the wet weight and organ coefficient of epididymis in ACN group were significantly lower (*P* < 0.05); after SP intervention, compared with ACN group, the wet weight and organ coefficient of epididymis in low SP intervention group were significantly higher (*P* < 0.05); the organ coefficient of epididymis in SP intervention group increased significantly (*P* < 0.05) (Tables 1 and 2).

### 3.2. Changes of Sperm Density in Rats

There was no significant difference in sperm density between groups (*P* > 0.05). Compared with the control group, the proportion of grade A and B sperm in ACN group increased significantly, and the proportion of grade D sperm decreased significantly(*P* < 0.05); after SP intervention, compared with ACN group, there was no significant difference in the proportion of sperm at all levels in low, medium, and high SP intervention groups (*P* > 0.05).

### 3.3. Changes of Sperm Motility Parameters in Rats

Compared with the control group, the sperm VCL, VSL, VAP, and mad in ACN group increased significantly, and the BCF decreased significantly (*P* < 0.05); after AP intervention, compared with ACN group, there was no significant difference in sperm motility parameters among low, medium, and high SP intervention groups (*P* > 0.05). See Figure 1.

### 3.4. Morphological Changes of Rat Testis

The pathological sections of testicular tissue of rats in each group were observed under light microscope. The seminiferous tubules in testicular tissue of rats in the control group were complete and closely arranged; spermatogenic cells at different developmental stages can be seen in the seminiferous tubules. Spermatogonia, primary spermatocytes, secondary spermatocytes, and spermatocytes can be seen from the basement membrane to the lumen. The cell layers are clear and orderly; mature sperm can be seen in the lumen; interstitial cells can be seen in groups between seminiferous tubules. In ACN group, the seminiferous tubules were atrophic and deformed, and the diameter of seminiferous tubules became smaller; the number of spermatogenic cell layers decreased significantly, the number of primary spermatocytes and secondary spermatocytes decreased, and the number of mature sperms in the lumen was very small; the number of stromal cells decreased. In the low SP intervention group, only some seminiferous tubules were damaged, the number of spermatogenic cell layers and the number of mature sperms decreased; in the SP intervention group, the wall of spermatogenic tubules was relatively complete and arranged regularly, only a few layers of spermatogenic cells were reduced, and spermatogenic cells and mature sperm at all levels were seen in the lumen; in the high SP intervention group, the seminiferous tubules shrank and the diameter became smaller; the number and layers of spermatogenic cells decreased, the number of mature sperms decreased, and the number of stromal cells decreased.

### 3.5. Changes of Marker Enzymes in Rat Testis

Compared with the control group, the activities of AKP and SDH in testicular tissue of rats in ACN group decreased significantly (*P* < 0.05); after SP intervention, compared with ACN group, AKP activity increased significantly and LDH activity decreased significantly in low, medium, and high SP intervention groups (*P* < 0.05).

### 3.6. Expression Level of PI3K-NRF2/p38 Pathway-Related Genes

The results of RT-PCR showed that compared with the control group, the relative expression levels of PI3K, MKK7, JNK, and p38 mRNA in testis of rats in ACN group increased (*P* < 0.05); after SP intervention, compared with ACN group, the relative expression levels of MKK7, JNK, and p38 mRNA in testicular tissue of rats in low SP intervention group decreased (*P* < 0.05); the relative expression level of JNK mRNA in testicular tissue of rats in SP intervention group decreased (*P* < 0.05).

### 3.7. Expression Level of PI3K-NRF2/p38 Pathway-Related Proteins

Compared with the control group, the expression levels of PI3K, p-PI3K, MKK7, p-MKK7, JNK, p-JNK, p38, and p-p38 proteins and the ratios of p-JNK/JNK and p-p38/p38 increased in the testis of ACN group (*P* < 0.05); after SP intervention, compared with ACN group, the expression levels of PI3K, p-PI3K, MKK7, p-MKK7, JNK, p-JNK, p38, and p-p38 protein in testicular tissue of rats in low SP intervention group decreased, and the ratio of p-JNK/JNK and p-p38/p38 decreased (*P* < 0.05); the expression levels of PI3K, p-PI3K, MKK7, p-MKK7, JNK, p-JNK, p38, and p-p38 proteins and the ratio of p-PI3K/PI3K and p-JNK/JNK in testicular tissue of rats in middle SP intervention group decreased (*P* < 0.05); the ratios of p-PI3K/PI3K and p-JNK JNK in testicular tissue of rats in high SP intervention group decreased (*P* < 0.05).

## 4. Discussion

Sperm density, motility, and morphology are important indicators reflecting sperm quality. They can reflect the damage degree of exogenous chemicals to male reproductive system and evaluate male reproductive toxicity [10]. In this study, Casa system was used to analyze the quality of rat sperm. Casa system organically combines computer technology and advanced image processing technology. Through the observation of sperm movement, Casa system provides accurate data of various indexes of sperm quality and improves the detection speed and objectivity of results. This study found that the proportion of grade A and B sperms in ACN group increased significantly, the proportion of grade D sperm decreased significantly, and the sperm mobility and motility were significantly higher than those in the control group, suggesting that the increase of sperm motility may be caused by transient stress caused by short-term exposure to ACN [11]. There were no significant changes in sperm density, viability, and motility after SP intervention compared with ACN group, suggesting that SP had little effect on sperm density in this study, which may be related to the shorter action time [12].

Histopathological examination can reflect the damage of chemicals to target organs. It is one of the important items to evaluate the toxicity of exogenous chemicals. In this experiment, we observed that the seminiferous tubules in ACN group shrank and deformed, the number of stromal cells decreased, the layers of spermatogenic cells decreased and arranged disorderly, and the number of mature sperms in the lumen decreased [11]. The above situation of each dose of SP intervention group has been improved to a certain extent. The effect of low and medium SP intervention group is more obvious, which is similar to the result of organ coefficient, suggesting that SP has a certain protective effect on testicular injury induced by ACN. KP, ACP, LDH, and SDH are testicular marker enzymes, which play an important role in spermatogenesis and maturation, and are closely related to testicular function. AKP is mainly involved in the transport of nutrients in spermatogenic cells and is closely related to the proliferation and division of spermatogenic cells [13]. ACP is related to the degeneration of spermatogenic epithelium and the phagocytosis of testicular Sertoli cells. It mostly exists in the lysosome of Sertoli cells. It has the ability to remove damaged and aging cells. It plays an important role in maintaining the normal metabolism and physiological function of spermatogenic cells [14]. Its activity can be used as an indicator to measure whether spermatogenic disorder occurs. SDH mainly exists in the mitochondria of seminiferous tubules and spermatogenic cells. It provides energy for spermatogenic cells by catalyzing fructose into sorbitol. It plays an important role in sperm energy metabolism. Its activity can be used as an index to evaluate the function of sperm mitochondria. At the same time, it is also a marker enzyme for testicular pill maturity, sperm functional maturity, and perfect morphology. LDH belongs to glycolytic enzyme system, which is mainly distributed in seminiferous tubules and spermatogenic cells [15]. It participates in sperm energy metabolism and is also related to the maturation of spermatogenic epithelium. It is a marker enzyme of spermatogenic cell maturation. Xin et al. exposed male rats to ACN subchronic. The results showed that 10 mg/kg ACN could significantly increase the activity of LDH in testicular tissue and slightly increase the activities of AKP, ACP, and SDH. Then, with the increase of dose, the activities of LDH, ACP, and SDH in testicular tissue decreased [16]. The results showed that the activities of AKP and SDH decreased significantly in ACN group, indicating that ACN can affect the transport of testicular nutrients, interfere with testicular energy metabolism and the maturation of testicular spermatogenic epithelium, and cause a certain degree of damage to testis. After SP intervention, compared with ACN group, AKP activity increased significantly and LDH activity decreased significantly in low, medium, and high SP intervention groups, suggesting that SP can improve the above changes of testicular marker enzymes caused by ACN, that is, it can improve testicular energy metabolism and maturation of spermatogenic epithelium [17].

Under normal circumstances, oxidation and antioxidation in the body are in dynamic balance. When the free radicals produced by exogenous chemicals on the body exceed its scavenging capacity, it will lead to the excess of free radicals, the balance state will be broken, and the oxidative damage of cells and tissues will be caused [18]. ACN and its metabolite CEO can covalently combine with GSH to form adducts. At the same time, the released CN can induce the production of ROS, trigger free radical reaction, lipid peroxidation, and produce MDA and other active products. MDA is the product of lipid peroxidation. It has a strong toxic effect on the body. It can destroy the structure of biological macromolecules such as nucleic acid and protein [19]. It is an important physiological index of oxidative stress and lipid peroxidation. Sod can specifically scavenge O_2−_, inhibit oxygen free radical reaction and lipid peroxidation, and resist the damage caused by oxygen free radicals to cells. GSH is a kind of nonenzymatic small molecule antioxidant, which has the physiological functions of antioxidation, antiaging, and scavenging free radicals [20]. It can combine with the toxic compounds entering the body and urge them to be excreted from the body to neutralize the toxicity. GSH PX is an important peroxidase in the body. It can catalyze the reduction of toxic peroxides to nontoxic hydroxyl compounds and protect the structure and function of cell membrane from damage. Cat is a free radical scavenger and a marker enzyme of peroxisome. It can promote the decomposition of H_2_O_2_ into molecular oxygen and water, so as to protect tissues and cells from H_2_O_2_ damage [21]. T-AOC represents the comprehensive effect of enzymatic and nonenzymatic antioxidant capacity of the body, mainly reflects the dynamic balance of ROS in the internal environment, and is often used to evaluate the antioxidant capacity of the body. Zhao et al. found that after exposure to 50 mg/kg ACN for 13 weeks, the content of MDA in rat testis increased significantly and the activity of GSH PX decreased significantly. Under the experimental conditions, compared with the control group, the activity of GSH PX and the level of T-AOC in testicular tissue of ACN group decreased significantly, the content of MDA increased to a certain extent, and the content of GSH, the activity of SOD, and the level of cat decreased to a certain extent, suggesting that ACN leads to oxidative stress injury in testicular tissue of rats [22]. Some researchers found that SP can increase the activity of SOD in serum and GSH PX in the liver and reduce the content of MDA. Kilani et al. found that SP can significantly reduce MDA content and improve SOD activity and T-AOC level in hyperuricemia rats. Chen Junyi and others found that SP has a protective effect on lipid peroxidation and DNA damage of rat sperm caused by ACN [23]. 468 mg/kg SP can reduce ROS production, MDA content, SOD activity, and sperm DNA damage. The results showed that after SP intervention, compared with ACN group, the content of GSH and the level of T-AOC in testicular tissue in low SP intervention group were significantly increased, the content of MDA was reduced, and the activities of SOD, GSH PX, and cat were increased; in the SP intervention group, the content of MDA in testicular tissue decreased to a certain extent, and the content of GSH, the activity of SOD and cat, and the level of T-AOC increased to a certain extent, suggesting that SP can improve the oxidative stress of rat testicular tissue induced by ACN [24].

Oxidative stress can mediate the activation of many intracellular pathways, such as the study by MAPK et al. There are cross and feedback between these channels, which affect each other. MAPK is a kind of serine/threonine protein kinase, which can transmit exogenous signals down through multilevel protein kinase cascade reaction [25] and then regulate gene and cell physiological response to environmental changes. It exists widely in vivo. At present, four MAPK family members have been identified, namely, p38 MAPK, JNK, extracellular signal regulated kinase 1/2 (ERK1/2), and extracellular signal regulated kinase-5 (ERK5). They can play an important role in regulating cell growth, differentiation, and apoptosis. The MAPK signaling pathway is composed of three protein kinases, including MAP2K and MAP3K, which are associated with a variety of diseases, such as tumors, autoimmune diseases and diabetes, and developmental abnormalities [26]. When stimulated by growth factors, cytokines, or other factors, MAP3K-MAP2K-mapk phosphorylation is activated step by step. Serine/threonine residue phosphorylation of channel protein is the main way of MAPK pathway activation. Different exogenous stimuli activate different MAPK signaling pathways and then phosphorylate different downstream substrates, including various transcription factors and protein kinases, which eventually lead to a series of biochemical reactions such as cell proliferation, differentiation, and apoptosis [27]. PI3K is a member of MAP3K family. It is ROS sensitive and is the key in oxidative stress-mediated apoptosis. After oxidative stress, the Thr 845 site of PI3K is phosphorylated and then activated. Activated PI3K can phosphorylate downstream MKK4 and MKK7. Activated MKK4 and MKK7 activate JNK by phosphorylating Thr 183 and Tyr 185. They can also phosphorylate downstream MKK3 and MKK6. Activated MKK3 and MKK6 activate p38 by phosphorylating Thr 180 and Tyr 182. The results of this study showed that compared with the control group, the relative expression levels of PI3K, MKK7, JNK, and p38 mRNA, the expression levels of PI3K, p-PI3K, MKK7, p-MKK7, JNK, p-JNK, p38, and p-p38 protein, and the ratio of p-JNK/JNK and p-p38/p38 increased in ACN group; after SP intervention, compared with ACN group, the relative expression levels of MKK7, JNK, and p38 mRNA, the expression levels of PI3K, p-PI3K, MKK7, p-MKK7, JNK, p-JNK, p38, and p-p38 protein and the ratio of p-JNK/JNK and p-p38/p38 decreased in low SP intervention group [28]; The relative expression level of JNK mRNA, the expression level of PI3K, p-PI3K, MKK7, p-MKK7, JNK, p-JNK, p38, and p-p38 protein and the ratio of p-PI3K/PI3K and p-JNK/JNK decreased in the middle SP intervention group. The ratio of p-JNK/JNK and p-p38/p38 in testicular tissue of rats in high SP intervention group decreased, suggesting that SP can inhibit the activation of PI3K-NRF2/p38 signal pathway induced by ACN.

In conclusion, SP can reduce ACN induced testicular oxidative stress, inhibit the activation of PI3K-NRF2/p38 signaling pathway, and then inhibit mitochondrial mediated apoptosis. This study detected the related indicators of testicular oxidative stress and speculated that SP may play a protective role by reducing oxidative stress, but ROS was not detected and there was no direct evidence. Therefore, ROS level should be detected in future research. In this study, SP intervention can improve the sperm quality and testicular injury induced by ACN, but the changes of various indexes after different doses of SP intervention do not show consistent results. In future research, we can refine the grouping and explore the best dose of SP for the protection of ACN reproductive injury.

## Figures and Tables

**Figure 1:** Changes in sperm motility parameters in rats.

**Figure 2:** Changes in the tissue morphology of the testis in rats.

**Figure 3:** Changes in the rat testis marker enzymes.

**Figure 4:** Expression levels of genes associated in the PI3K 1-NRF2/p38 pathway.

**Figure 5:** The protein expression levels associated with the PI3K-NRF2 pathway.

**Table 1:** General condition and organ coefficient changes in rats.

Group	Weight (g)	Orchis		Epididymis	
		Wet weight (g)	Organ coefficient	Wet weight (g)	Organ coefficient
NC	349.64 ± 24.20	3.15 ± 0.23	0.92 ± 0.07	1.11 ± 0.07	0.33 ± 0.04
ACN	333.64 ± 20.14	2.99 ± 0.15	0.91 ± 0.05	0.99 ± 0.07	0.31 ± 0.02
Low	329.41 ± 18.47	3.04 ± 0.28	0.93 ± 0.09	1.05 ± 0.05	0.33 ± 0.03
Middle	315.63 ± 13.87	3.08 ± 0.21	0.99 ± 0.10	0.99 ± 0.06	0.34 ± 0.04
High	312.54 ± 14.02	2.90 ± 0.56	0.93 ± 0.03	0.95 ± 0.15	0.31 ± 0.05

**Table 2:** Changes in sperm density in rats.

Group	Sperm density	Sperm movement mode			
		A level	B level	C level	D level
NC	5.73 ± 1.19	6.02 ± 2.14	11.46 ± 2.98	40.31 ± 2.58	42.31 ± 4.78
ACN	6.68 ± 2.48	12.34 ± 3.52	15.64 ± 4.20	42.12 ± 4.69	29.321 ± 8.15
Low	6.39 ± 2.87	10.57 ± 4.79	14.24 ± 4.58	42.64 ± 5.80	32.64 ± 10.42
Middle	5.97 ± 2.45	10.54 ± 4.25	14.79 ± 1.35	42.43 ± 6.25	32.65 ± 8.12
High	5.96 ± 1.42	10.53 ± 3.25	14.98 ± 2.31	43.12 ± 4.02	31.58 ± 5.61

## Data Availability

No data were used in this study.
